# Human Resource Planning and Configuration Based on Machine Learning

**DOI:** 10.1155/2022/3605722

**Published:** 2022-03-15

**Authors:** Shuai Yuan, Qian Qi, Enliang Dai, Yongfeng Liang

**Affiliations:** ^1^School of Management Engineering and Business, Hebei University of Engineering, Handan 056000, China; ^2^School of Artificial Intelligence, Beijing University of Posts and Telecommunications, Beijing 100000, China; ^3^School of Labor and Human Resources, Renmin University of China, Beijing 100000, China; ^4^Beijing Miss Fresh E-Commerce Co. Ltd, Beijing 100000, China

## Abstract

Human resources are the core resources of an enterprise, and the demand forecasting plays a vital role in the allocation and optimization of human resources. Starting from the basic concepts of human resource forecasting, this paper employs the backpropagation neural network (BPNN) and radial basis function neural network (RBFNN) to analyze human resource needs and determine the key elements of the company's human resource allocation through predictive models. With historical data as reference, the forecast value of current human resource demand is obtained through the two types of neural networks. Based on the prediction results, the company managers can carry out targeted human resource planning and allocation to improve the efficiency of enterprise operations. In the experiment, the actual human resource data of a certain company are used as the experimental basic samples to train and test the two types of machine learning tools. The experimental results show that the method proposed in this paper can effectively predict the number of personnel required and can support the planning and allocation of human resources.

## 1. Introduction

Human resources are valuable corporate resources and are of great significance to their predictive analysis. Many experts and scholars all over the world have conducted relevant research studies [1–4]. Human resource demand forecasting generally needs to follow the principle of correlation and the principle of inertia. The principle of correlation is based on the correlation between the research objects and uses other objects to predict the targeted object [5–12]. For example, there is a clear correlation between A, B, and C. In the research process, rich data of A, B, and C can be obtained. At the same time, the trend value of B and C can be predicted by suitable forecasting methods, and finally the correctness can be achieved by making predictions based on A. The principle of inertia specifically refers to the slow progress of A or its regular development, and some valid past data can be obtained. Under this premise, you can choose appropriate means to predict the trend value of A. The human resource demand forecasting model is mainly based on qualitative and quantitative analysis. Qualitative analysis methods mainly include the Delphi method, subjective judgment method, microintegration method, and so on. The above methods rely more on experts or experienced people, and they all have the disadvantage of subjective components. As a result, the prediction results are prone to be non-consensual judgments. The quantitative analysis methods mainly include the production function method, ratio method, trend method, regression analysis method, and so on. The above quantitative analysis is based on the existing data for predictive analysis. The prediction logic is rigorous and overcomes the shortcomings of qualitative methods. However, there are also problems such as low prediction accuracy and difficulty in collecting data. Therefore, the combination of quantitative and qualitative methods has naturally become the research direction of enterprise human resource forecasting [13–17].

Zhandong and Chi [18] used the Delphi method to study the human resource forecasting of enterprises and explained the importance of human resource forecasting in enterprise management. Belhaj et al. [1] used the Markov model to predict the human resources of the enterprise and obtained the demand for the human resources of the enterprise in the future [19]. Wu and Nagahashi [20] used the grey forecasting model to carry out human resource forecasting analysis for enterprises, which provided a reference for its human resource planning. Qu et al. [21] predicted the human resources of enterprises based on backpropagation neural network (BPNN) and believed that network can obtain better prediction results. There are many factors affecting human resource demand and non-linear correlation. At the same time, traditional analysis and forecasting methods such as the analytic hierarchy process, multiple linear regression method, and Delphi method have shortcomings and shortcomings such as low prediction accuracy and biased subjective analysis. Therefore, common predictive analysis methods cannot truly reflect the nature of the problem. As a remedy, researchers began to study prediction methods based on machine learning models, which have higher superiority compared with traditional prediction methods [21–25]. Common modern machine learning methods include BPNN, K-nearest neighbors (KNN), support vector machine (SVM), and so on. In addition, the machine learning methods based on tree models were also widely used for data prediction, such as basic decision tree models and related integrated models such as random forests. Therefore, the research on human resource forecasting using machine learning plays an important role in improving forecasting accuracy [26–30].

This paper studies the method of personnel resource planning and allocation based on machine learning. The basic idea of this method is to use machine learning algorithms to predict enterprise human resource needs and dynamically adjust staffing accordingly. Specifically, this paper uses two machine learning models, BPNN and radial basis function neural network (RBFNN). Both types of models are based on neural networks, and robust model parameters are obtained by optimizing training algorithms. For the company's human resource needs, the historical data are used as training samples to train the two models to obtain a robust prediction model. Finally, the corresponding predicted value of human resource demand can be obtained under current conditions, which can be used as a reference for enterprise management personnel in personnel planning and configuration. The experiment uses human resource data of a certain company as the samples. Also, the validity of the proposed method can be verified according to the experimental results.

## 2. Machine Learning Models

### 2.1. BPNN

BPNN is a kind of multilayer feedforward neural network with signal forward transmission and error backward propagation [11–15]. It is widely used in the fields of function approximation and pattern recognition. The topological structure of BPNN includes input layer, hidden layer, and output layer, and each layer is composed of neuron connections. In the forward calculation process of the BPNN, information is input by the input layer and processed and calculated by the hidden layers, and the output layer outputs the processing results. In the backward propagation of the error, the error of the processing result of the output layer is calculated. The error signal is propagated back, and the weight of the connection between each neuron is corrected by the method of gradient descent, so as to realize the network optimization.

The training of BPNN includes two processes: forward propagation of signal and backward feedback of error. The forward propagation means that in the calculation, the signal enters the hidden layer after parallel weighting calculation from the input layer and then enters the output layer through weighting processing to obtain the output. The direction of the reverse feedback process is carried out from output to input. The weights and thresholds are adjusted according to the actual error. Through continuous repetition of forward calculation and reverse feedback, the output result can finally meet the requirements. A basic model of BPNN is shown in Figure 1. In this figure, (*x*_1_, *x*_2_,…, *x*_*j*_,…, *x*_*m*_) is the input quantity, and the subscript is the input quantity number, which corresponds to the input layer node; (*y*_1_, *y*_2_,…, *y*_*k*_,…, *y*_*t*_) is the output quantity, and the subscript is the output quantity number, which corresponds to the output layer node; (*θ*_1_, *θ*_2_,…, *θ*_*i*_,…, *θ*_*q*_) are the thresholds introduced for the hidden layer, and the subscript is the hidden node number; there may be multiple hidden layers in the neural network; (*a*_1_, *a*_2_,…, *a*_*k*_,…, *a*_*t*_) are the threshold values introduced for the output layer, and the subscript is the output node number. There is only one output layer in the neural network; *ε* denotes the error value.

In the process of forward propagation, the input *n*_*i*_ and output *o*_*i*_ of the *i*th node in the hidden layer can be calculated as follows:

(1) $$\begin{array}{c} n_{i}=\sum_{j=1}^{m}w_{ij}x_{j}+\theta_{i},\\ o_{i}=\phi \left({\text{net}}_{i}\right)=\phi \left(n_{i}\right). \end{array}$$

In the process of forward propagation, the input net_*k*_ and output of the *k*th in the output layer are calculated as follows:

(2) $$\begin{array}{c} {\text{net}}_{k}=\sum_{u=1}^{q}w_{ki}o_{i}+a_{k}=\sum_{u=1}^{q}w_{ki}\phi \left(\sum_{j=1}^{m}w_{ij}x_{j}+\theta_{i}\right)+a_{k},\\ {\text{out}}_{k}=\psi \left({\text{net}}_{k}\right), \end{array}$$

where *w*_*ij*_ is the weight of the *j*th input variable at the *i*th node of the hidden layer; *ϕ* is the activation function of the hidden layer; and *ψ* is the activation function of the output layer. In order to enhance the large-scale non-linear fitting ability, according to actual use experience, the hidden layer activation function selects the bipolar S-shaped tansig function, and the output layer activation function selects the linear purelin function.

The error function *E*_*P*_ of the *P*th sample is shown in equation (3), where *T*_*k*_ is the expected output value of the *k*th node.

(3) $$\begin{array}{c} E_{P}=\frac{1}{2}\sum_{k=1}^{1}{\left(T_{k}-{\text{out}}_{k}\right)}^{2}. \end{array}$$

The total error *E* of *P* training samples is

(4) $$\begin{array}{c} E=\frac{1}{2}\sum_{p=1}^{P}\overset{l}{\underset{k=1}{\sum }}{\left(T_{k}^{P}-{\text{out}}_{k}^{P}\right)}^{2}. \end{array}$$

In the feedback process, the weight correction amount and threshold correction amount of the hidden layer and the output layer can be written as

(5) $$\begin{array}{c} \Delta w_{ij}=-\eta \frac{\partial E}{\partial w_{ij}},\Delta \theta_{i}=-\eta \frac{\partial E}{\partial \theta_{i}},\\ \Delta w_{kj}=-\eta \frac{\partial E}{\partial w_{kj}},\Delta a_{k}=-\eta \frac{\partial E}{\partial a_{k}}, \end{array}$$

where *η* is the coefficient determining adjustment rate.

The specific steps of BPNN are as follows:

  Step 1: Network initialization: the necessary network parameters are determined. Generally, there are the number of input layer nodes, the number of hidden layer nodes, the number of output layer nodes, connection weights and thresholds, transfer function types, and so on.
  Step 2: According to the parameters determined in Step 1, the hidden layer output calculation is carried out.
  Step 3: Same as above, the input calculation of the output layer is carried out.
  Step 4: The network error is calculated as follows: the expected output-network predicted output.
  Step 5: The connection weight and threshold are updated according to the network error and network learning rate.
  Step 6: The judgment is made on whether the algorithm is terminated. If it is not over, return to Step 2 to continue network training.

It should be noted that there are many kinds of transfer functions, and the threshold transfer function (Hardlim) is generally used. The second is that the network data need normalized data during the training process, which requires that the data are normalized to (0, 1). Also, the data are restored when the data are output. Third, in general, the number of hidden layer nodes needs to be determined manually. Set the number of input layer nodes to be *n*, the number of hidden layer nodes to be *l*, and the number of output layer nodes to be *m*, and they satisfy the following relationship:

(6) $$\begin{array}{c} \left\{\begin{array}{c} l<n-1,\\ l<\sqrt{m+n}+a,\left(0<a<10\right),\\ l=\log_{2}\;n. \end{array}\right.. \end{array}$$

### 2.2. RBFNN

Furthermore, because the BPNN generally needs to iteratively determine the connection weights, a relatively large time delay will be generated for a large amount of data processing [16–20]. The RBFNN obtains a value by calculating the norm of the input sample and the hidden layer point (center point) and substituting it into the radial basis function (Gaussian function, quadratic function, inverse quadratic function, and so on). After the weights are multiplied and added, the corresponding output is obtained. The network is simple, and the learning convergence speed is faster, which can make up for the deficiencies of BPNN.

RBFNN is a three-layer forward network, and its network structure is shown in Figure 2. Among them, *W*_1_ and *b*_1_ are the connection weight matrix and bias vector from the input layer to the hidden layer. *W*_2_ and *b*_2_ are the connection weight matrix and the connection weight matrix from the hidden layer to the output layer. The input layer is composed of signal nodes, and the number of neurons is the dimension of the input sample. The activation function of the hidden layer neurons is a RBF that is radially symmetric and attenuated to the center point and is commonly used as Gauss function, reflected sigmoidal function, inverse multiquadric function, etc. The output layer responds to the input pattern, and the number of neurons is equal to the dimension of the output sample. The transformation from the input space to the hidden layer space is non-linear, and the transformation from the hidden layer space to the output layer space is linear, so the mapping of RBFNN from input to output is also non-linear.

The basic idea of RBFNN is to use RBF as the activation function of the hidden layer neurons to form the hidden layer space, so that the input vector can be directly mapped to the hidden layer space. Also, the mapping from the hidden layer space to the output layer space is linear, that is, the network output of RBFNN is the linear weighted sum of the output of hidden layer neurons. The connection weight from the hidden layer to the output layer is an adjustable parameter of RBFNN. It can be seen that although the network input to output mapping is non-linear, the network output is linear for the adjustable parameters, so the adjustable parameters of the network can be solved directly by linear equations, which greatly accelerates the learning speed and avoids the local minima problems. RBFNN is a function approximation network that non-linearly maps the input space to the output space. The weight vector of the array beam design is a non-linear function of the position of the array element, so the use of RBFNN can realize the mapping from the position of the array element to the weight vector of the array.

According to the above discussion, the overall expression of RBFNN is

(7) $$\begin{array}{c} f\left(x\right)=\omega_{0}+\sum_{i=1}^{n}\omega_{i}\varphi \left(\left\|x-c_{i}\right\|\right), \end{array}$$

where *ω* is the connection weight, which can be iteratively obtained by the least squares method, and the calculation formula is

(8) $$\begin{array}{c} \omega =\exp\left(\frac{h}{c_{\max}^{2}}{\left\|x_{p}-c_{i}\right\|}^{2}\right),\;i=1,2,\ldots ,h,p=1,2,\ldots ,P. \end{array}$$

The specific learning algorithm steps are as follows:

  Step 1: The K-means clustering method is used to solve the center of the radial basis function; generally, after the network initialization, the input data are calculated according to the nearest neighbor rule, and grouping and re-adjusting the clustering center are completed in 3 steps.
  Step 2: The variance of RBF of the RBFNN is calculated.
  Step 3: The least squares algorithm is employed to calculate the weight between the hidden layer and the output layer.

## 3. Experiment and Analysis

### 3.1. Dataset and Comparison Method

Taking a company's personnel data as an example, the original data (2009–2020) are divided into two parts. The first 10-year data are the basic data, and the 11th year data are the verification data, and the model is trained and solved. When judging the pros and cons of different models' predictive performance, some quantitative index systems are needed. According to the existing literature, this paper selects three indicators: mean squared error (MSE), mean absolute percentage error (MAPE), and symmetric mean absolute percentage error (SMAPE), as the evaluation indexes for the predictive performance. The specific calculation formulas of the above three error indicators are as follows:

(9) $$\begin{array}{c} \text{MSE}=\frac{1}{N}\sum_{\tau =t_{0}}^{t_{N-1}}{\left(y_{\tau }-y_{\tau }^{0}\right)}^{2},\\ \text{MAPE}=\frac{100\text{\%}}{N}\sum_{\tau =t_{0}}^{t_{N-1}}\left|\frac{y_{t}-y_{t}^{0}}{y_{t}^{0}}\right|,\\ \text{SMAPE}=\frac{100\text{\%}}{N}\sum_{\tau =t_{0}}^{t_{N-1}}\frac{\left|y_{t}-y_{t}^{0}\right|}{\left(\left|y_{t}\right|+\left|y_{t}^{0}\right|\right)/2}. \end{array}$$

## 4. Results and Analysis

In addition to the two models used in this paper, two traditional methods from the literature [12, 18] are also selected for comparative analysis in the experiment. Taking selected experimental data as samples, based on the three indicators of MSE, MAPE, and SMAPE to test different methods, the statistics of the results of different methods are shown in Table 1. It can be seen that the overall performance of the BPNN and RBFNN selected in this paper is better than that of the two traditional methods, reflecting the performance advantages of the machine learning models. Comparing BPNN and RBFNN, the latter has more advantages in overall performance because of the consideration of non-linear factors.

In the actual process, due to the influence of external factors such as market changes and changes in the international situation, the prediction model may have certain deviations. For this reason, this paper applies a certain degree of noise conditions to the experimental data to reflect the influence of external influences on the allocation of human resources. On this basis, the performance trend of various methods is tested using MSE as the basic evaluation index, and the results are shown in Figure 3. It can be seen from the figure that the performance of various methods is degraded to a certain extent due to the influence of noise. As the signal-to-noise ratio (SNR) decreases, the MSE keeps increasing. In comparison, the two models used in this paper can maintain the best prediction performance under different noise interference conditions, which further enhances its performance advantages. Comparing BPNN and RBFNN, the latter has better overall noise robustness due to the consideration of the possible non-linear effects of noise.

## 5. Conclusion

The sustainable demand forecast of human resources is the prerequisite and basis for the correct deployment of personnel planning. This paper proposes a human resource prediction method based on machine learning to address the above problems. Two types of neural networks, BPNN and RBFNN, are used to predict the human resource needs of enterprises. We train the two types of models based on the historical data of human resources to obtain predictive models. According to the current enterprise situation, the current enterprise human resource forecast value can be obtained. In the experiment, the two models are tested and verified using human resource data of a certain enterprise. The experimental results show that the proposed method is effective for enterprise personnel resource forecasting and can support enterprise managers to carry out scientific personnel planning and allocation.

## Figures and Tables

**Figure 1:** Basic structure of BPNN.

**Figure 2:** Basic structure of RBFNN.

**Figure 3:** Performance measured by MSE achieved by different methods under noises.

**Table 1:** Comparison of different methods in the prediction of human resources.

Method	Evaluation index		
	MSE	MAPE	SMAPE
BPNN	0.32	0.43%	0.43%
RBFNN	0.41	0.47%	0.46%
Comparison 1	0.45	0.52%	0.57%
Comparison 2	0.47	0.54%	0.52%

## Data Availability

The dataset used to support the findings of this study is available from the corresponding author upon request.
